# lncRNA lnc-TSI Inhibits Metastasis of Clear Cell Renal Cell Carcinoma by Suppressing TGF-β-Induced Epithelial-Mesenchymal Transition

This article has been retracted.

**DOI:** 10.1016/j.omtn.2020.08.003

**Published:** 2020-08-05

**Authors:** Peng Wang, Weixiong Chen, Tongtong Ma, Zhaoyu Lin, Chongbin Liu, Youhua Liu, Fan Fan Hou

**Affiliations:** 1 Division of Nephrology, Nanfang Hospital, Southern Medical University, State Key Laboratory of Organ Failure Research, National Clinical Research Center of Kidney Disease, Guangzhou 510515, China; 2 Department of Stomatology, Longgang District Central Hospital, Affiliated to Guangzhou University of Traditional Chinese Medicine, Shenzhen, Guangdong 518116, China; 3 Department of Anesthesiology, The First Affiliated Hospital of Guangzhou Medical University, Guangzhou 510120, China; 4 Guangdong Provincial Key Laboratory of Malignant Tumor Epigenetics and Gene Regulation, Sun Yat-sen Memorial Hospital, Sun Yat-sen University, Guangzhou 510120, China; 5 Department of Oral & Maxillofacial Surgery, Sun Yat-sen Memorial Hospital, Sun Yat-sen University, Guangzhou 510120, China; 6 Guangzhou Regenerative Medicine and Health Guangdong Laboratory, 510005 Guangzhou, China

**Keywords:** clear cell renal cell carcinoma, long noncoding RNA, metastasis, TGF-β signaling

## Abstract

The transforming growth factor-β (TGF-β)/Smads signal plays an important role in cancer metastasis by mediating the epithelial-mesenchymal transition (EMT) in cancer cells. lnc-TSI is a recently identified long noncoding RNA that negatively regulates the TGF-β/Smads signal. The present study was conducted to test the hypothesis that lnc-TSI inhibits metastasis in clear cell renal cell carcinoma (ccRCC) by regulating the TGF-β/Smad3 pathway. Herein, we show that lnc-TSI was upregulated in ccRCC cells and tissue and was associated with activation of the TGF-β/Smads signal. Depleting lnc-TSI enhanced tumor cell invasion and metastasis *in vitro* and ccRCC lung metastasis *in vivo*, whereas overexpressing lnc-TSI inhibited ccRCC cell invasion and tumor metastasis. Mechanistic studies indicated that lnc-TSI specifically inhibited the phosphorylation of Smad3 and subsequent EMT by binding with the MH2 domain of Smad3 to block the interaction between Smad3 and TGF-β receptor I in ccRCC cells. In a cohort of 150 patients with ccRCC, expression of lnc-TSI in tumors was negatively correlated with phosphorylated (p)Smad3 and activated EMT markers. Patients with expression of tumor lnc-TSI greater than or equal to the median at radical nephrectomy had a higher survival rate compared to those with lnc-TSI below the median during follow-up. These findings reveal a new regulatory mechanism of ccRCC metastasis and suggest a potential molecular target for the development of anti-cancer drugs.

## Teaser

TGF-β/Smad3 signaling has been found to play an important role in cancer metastasis. Wang et al. show that lncRNA lnc-TSI inhibits cancer cell invasion and tumor metastasis via specifically inhibiting the phosphorylation of Smad3 and subsequent EMT, which could be potentially applied in treatments for cancer metastasis.

## Introduction

Renal cell carcinoma (RCC) remains one of the most commonly diagnosed carcinomas in humans, with constantly rising mortality.^1^^,^^2^ Clear cell RCC (ccRCC), which comprises 75%–80% of RCCs, is not sensitive to radiotherapy or chemotherapy.^3^ Although it is treatable by surgery, the recurrence rate is still up to 20%–40% after radical nephrectomy, and hence the 5-year survival rate of ccRCC was only 20% after surgical resection.^4^^,^^5^ Therefore, it is of importance to understand the underlying mechanisms for the metastasis of ccRCC to identify new therapeutic strategies.

The epithelial-mesenchymal transition (EMT), which is comprised of multiple dynamic transitional states between epithelial and mesenchymal phenotypes, plays a critical role in regulation of progression and metastasis in many types of tumors, including ccRCC.^6^, ^7^, ^8^ Emerging evidence has shown that EMT was highly modulated by a number of transcription factors and regulators.^9^, ^10^, ^11^ In particular, transforming growth factor-β (TGF-β)/Smads signaling, a crucial driver of EMT, plays a pivotal role in cancer progression, migration, invasion, and metastasis.^12^, ^13^, ^14^ TGF-β initiates its molecular functions by binding with the TGF-β type II receptor, which phosphorylates the TGF-β type I receptor (TβRI), resulting in the phosphorylation of Smad3 and Smad2 and the following nucleus translocation of Smad2, Smad3, and Smad4.^15^^,^^16^ The phosphorylation of Smad3 by TβRI was a key initial event in the activation of TGF-β/Smads signaling.^17^, ^18^, ^19^ Despite the importance of the TGF-β-induced EMT, as a regulator of tumor metastasis, the molecular mechanisms underlying EMT in ccRCC have not been completely understood.

We recently identify a poorly conserved and kidney-enriched long noncoding RNA (lncRNA), which we termed TGF-β/Smad3-interacting lncRNA (lnc-TSI).^18^ lnc-TSI is specifically expressed in human tubular epithelial cells and acts by binding with the MH2 domain of Smad3, blocking the interaction of Smad3 with TβRI and inhibiting renal fibrogenesis.^18^ Given that ccRCC is a malignant tumor that originates from the renal parenchyma urinary tubule epithelial system, we therefore hypothesized that lnc-TSI may regulate EMT in ccRCC cells via suppressing the TGF-β/Smad3 pathway.

In this study, we investigated the potential role of lnc-TSI involved in the invasion, migration, and metastasis of ccRCC and its underlying mechanisms. We demonstrated for the first time that lnc-TSI inhibited the metastasis of ccRCC via inhibition of the phosphorylation of Smad3 and the subsequent EMT. This discovery adds to our understanding of the complex regulation of EMT in ccRCC and provides a potential new therapeutic target for this malignant tumor.

## Results

### TGF-β1/Smad3 Signaling Is Activated in ccRCC Cells and Tissue

Data from the GEO ccRCC patient datasets GEO: GSE14994 (n = 37) and GSE6344 (n = 20) were downloaded and analyzed for the expression of TGF-β1 mRNA. TGF-β1 transcription was upregulated in ccRCC tissue compared to that in renal tissue from normal subjects (Figures 1A and 1B). In a tissue microarray study, overexpression of TGF-β1 and phosphorylated (p)Smad3 were observed in ccRCC tissue but not in normal tissue adjacent to the tumor (Figure 1C).

**Figure 1:** lnc-TSI Was Upregulated in ccRCC Cells and Was Transcribed by Smad3 (A and B) GEO datasets revealed upregulation of TGF-β1 mRNA in human ccRCC tissues GEO: GSE14994 (n = 37, A) and GEO: GSE6344 (n = 20, B). (C) Immunohistochemistry results indicated that TGF-β and pSmad3 were upregulated in ccRCC tissues compared to adjacent tissues. (D) Representative images of Transwell assays (D_1_) and the data analysis results (D_2_) showed that TGF-β1 enhanced cell invasiveness in ccRCC cells. (E) Representative images of Caki-1 and 786-O cells treated with TGF-β1 (10 ng/mL) for 72 h. Cells became elongated and spindle-like phenotypes after exposure to TGF-β1. Scale bar represents 50 μm. (F) Western blot analysis and quantitative data of E-cadherin, N-cadherin, Vimentin, and Snail protein levels in TGF-β1 (10 ng/mL)-stimulated 786-O and Caki-1 cells. (G and H) qRT-PCR assay (G) and northern blot (H) showed that lnc-TSI was upregulated in Caki-1 and 786-O cells compared to normal human tubular epithelial cell (HK2) and that lnc-TSI expression was upregulated upon TGF-β1 stimulation. (I) RT-PCR showing lnc-TSI expression in the cytoplasm (cyto.) and nuclear (nu.) fractions of Caki-1 cells treated with TGF-β1 (10 ng/mL, 24 h). (J) Confocal FISH images showing cytoplasmic localization of lnc-TSI in 786-O and Caki-1 cells. U6 small nu. RNA was detected as control. (K) Luciferase reporter assays showed that knocking down Smad3 decreased the transcription activity of lnc-TSI. (L) Western blot analysis of Smad3 protein level after immunoprecipitation and ChIP assay showed that Smad3 occupied at the lnc-TSI promoter in Caki-1 cells. Data are expressed as means ± SD of three independent experiments. ∗p < 0.05, ∗∗p < 0.01, ∗∗∗p < 0.001.

To evaluate the effect of TGF-β1 on ccRCC cells, we incubated ccRCC cell lines (786-O and Caki-1) with TGF-β1. Cells exposed to TGF-β1 showed increased invasiveness (Figure 1D) and presented a spindle-like phenotype change (Figure 1E) with decreased expression of E-cadherin and increased expression of N-cadherin, Vimentin, and Snail (Figure 1F).

### lnc-TSI Is Upregulated in ccRCC Cells and Transcribed by Smad3

The expression levels of lnc-TSI in ccRCC cell lines (Caki-1 and 786-O) were significantly upregulated as compared to a normal human tubular epithelial cell line (HK2) (Figures 1G and 1H). Real-time PCR of the nuclear and cytoplasmic fractionations further demonstrated that lnc-TSI was predominantly localized in the cytoplasm of ccRCC cells (Figure 1I), which was verified by a fluorescence *in situ* hybridization (FISH) assay (Figure 1J).

Furthermore, knockdown of Smad3 significantly reduced lnc-TSI promoter activity (Figure 1K). Chromatin immunoprecipitation (ChIP) analysis with an anti-Smad3 antibody found that Smad3 was occupied at the lnc-TSI promoter in ccRCC cells (Figure 1L). These results indicated that lnc-TSI was transcribed by Smad3.

### lnc-TSI Inhibits Smad3 Phosphorylation in ccRCC Cells

Our previous study showed that lnc-TSI inhibits TGF-β1 signaling by specifically hindering the phosphorylation of Smad3 in tubule epithelial cells.^18^ To investigate whether lnc-TSI has an effect in ccRCC cells, we knocked out or overexpressed lnc-TSI in ccRCC cells (Figures S1A–S1C). Knocking out lnc-TSI in both Caki-1 (Figure 2A) and 786-O cells (Figure S1D) significantly enhanced the expression of pSmad3 but not total Smad3, pSmad2, or total Smad2. However, overexpressing lnc-TSI remarkably reduced the phosphorylation of Smad3 in ccRCC cells (Figure 2B; Figure S1E). Given the off-target effects of CRISP-Cas9 technology, we validated the effect of lnc-TSI on the TGF-β1-induced Smad3 phosphorylation using a second small guide RNA (sgRNA) clone (Figure S1F).

**Figure 2:** lnc-TSI Inhibited TGF-β1-Induced Smad3 Phosphorylation and nu. Translocation of the Smads Complex in Caki-1 Cells (A) Western blot showed that knocking out lnc-TSI promoted Smad3, but not Smad2, phosphorylation in Caki-1 cells in the presence or absence of exogenous TGF-β1 (A_1_). The data analysis results are shown in (A_2_) and (A_3_). (B) Western blot demonstrated that the overexpression of lnc-TSI inhibited Smad3, but not Smad2, phosphorylation in Caki-1 cells in the presence or absence of exogenous 10 ng/mL of TGF-β1 (B_1_). The data analysis results are shown in (B_2_) and (B_3_). (C) Immunofluorescence confocal images showed that knocking out lnc-TSI enhanced Smad3 nu. translocation in Caki-1 cells while overexpressing lnc-TSI inhibited Smad3 nu. translocation in the presence or absence of exogenous 10 ng/mL of TGF-β1 for 1 h (C_1_). The quantitative data of positive nu. Smad3 staining cells are shown in (C_2_). (D) Western blot in nucleus and cyto. of Caki-1 cells demonstrated that knockout of lnc-TSI promoted the nu. translocation of Smads in Caki-1 cells incubated with or without exogenous TGF-β1 (D_1_). β-Actin and lamin A/C were separately applied as the loading control for the cyto. or nucleus. The data analysis results are shown in (D_2_), (D_3_), and (D_4_). (E) Western blot demonstrated that the overexpression of lnc-TSI inhibited the nu. translocation of Smads in Caki-1 cells incubated with or without TGF-β1 (E_1_). The data analysis results are shown in (E_2_), (E_3_), and (E_4_). Data are expressed as means ± SD of three independent experiments. ∗p < 0.05, ∗∗p < 0.01, ∗∗∗p < 0.001.

Immunofluorescence staining showed that knocking out lnc-TSI increased Smad3 nuclear translocation, while forcing expression of lnc-TSI attenuated TGF-β1-induced Smad3 nuclear translocation in Caki-1 cells (Figure 2C). To further confirm the effect of lnc-TSI on Smads nuclear translocation, quantitative immunoblotting for nuclei or cytoplasm was conducted separately in TGF-β1-stimulated Caki-1 cells. The depletion of lnc-TSI enhanced Smad2, Smad3 and Smad4 nuclear translocation (Figure 2D), whereas overexpression of lnc-TSI inhibited the nuclear translocation of these Smads (Figure 2E).

### lnc-TSI Binds to the MH2 Domain of Smad3 and Inhibits the Interaction between TβRI and Smad3

To explore the molecular mechanism underlying the inhibition of Smad3 phosphorylation induced by lnc-TSI, we performed RNA pull-down assays *in vitro* followed by immunoblotting assays. The results showed that lnc-TSI specifically bound with Smad3, but not with other TGF-β1 signaling-related proteins, such as SARA, Smad2, Smad4, Smad7, and TβRI (Figure 3A). Immunofluorescence of Smad3 showed co-localization of lnc-TSI with Smad3 in the cytoplasm of TGF-β1-stimulated ccRCCs (Figure 3B). An RNA pull-down assay with Caki-1 cells transfected with full-length or truncated Smad3 mutations showed that lnc-TSI could directly bind to the MH2 domain of Smad3 (Figures 3C and 3D). Co-immunoprecipitation (coIP) assays showed that knockout of lnc-TSI increased the interaction between TβRI and Smad3 in the presence or absence of exogenous TGF-β1 (Figure 3E), while overexpression of lnc-TSI hindered this interaction (Figure 3F), suggesting that lnc-TSI inhibited Smad3 phosphorylation via binding with the MH2 domain of Smad3 and therefore inhibits the interaction between TβRI and Smad3. To identify the nucleotide (nt) sequence of lnc-TSI that binds Smad3, we constructed a series of lnc-TSI deletion mutants. RNA pull-down assays showed that the mutants containing nt 301–450 of lnc-TSI bound with Smad3 comparable to that of full-length lnc-TSI, which suggested that nt 301–450 represent the functional region for the interaction of lnc-TSI with Smad3 (Figure 3G). According to the RNAfold package, there were two stem-loop structures folded by nt 301–450 of lnc-TSI, termed stem-loop A and stem-loop B (Figure 3H).^20^ Deletion mutation of either stem-loop A or stem-loop B completely suppressed the binding of lnc-TSI with Smad3 (Figure 3I), indicating that stem-loop A and B were the regions where lnc-TSI bound with Smad3. Furthermore, incubation of the lnc-TSI complementary sequence with biotinylated lnc-TSI at different molar ratios in advance decreased the interaction between lnc-TSI and Smad3 in a dose-dependent manner (Figure 3J).

**Figure 3:** lnc-TSI Bound to Smad3 and Blocked the Interaction between TβRI and Smad3 in ccRCC Cells (A) lnc-TSI bound to Smad3 in Caki-1 cell lysates as shown by western blot after RNA pull-down. (B) Confocal images showed the colocalization of lnc-TSI and Smad3 in Caki-1 cells stimulated with TGF-β1 (10 ng/mL) for 24 h. (C) To test the binding domain of Smad3 with lnc-TSI, deleted mutants of Smad3 fragments were constructed and labeled by FLAG. (D) Western blot after RNA pull-down showed that lnc-TSI interacted with the MH2 domain and the full length of Smad3 in Caki-1 cell lysates. (E) Cell lysates of Caki-1 cells with lnc-TSI knockout or control were immunoprecipitated (IP) with anti-Smad3 antibody followed by immunoblotting (IB). Representative images (E_1_) and data analysis (E_2_) showed that knockout of lnc-TSI increased the interaction between Smad3 and TβRI. Whole-cell lysates (WCLs) were used as controls. (F) Representative images (F_1_) and data analysis (F_2_) showed that overexpressing lnc-TSI decreased the interaction of Smad3 with TβRI. (G) RNA pull-down showing the interaction of lnc-TSI mutants with Smad3 *in vitro*. (H) According to the RNAfold package, lnc-TSI was predicted to form two stem-loop structures with nucleotides (nt) sequence 301–450. (I) RNA pull-down indicated that deletion mutations of either stem-loop A or stem-loop B abolished the binding capacity of lnc-TSI to Smad3. (J) RNA pull-down indicated that preincubating lnc-TSI with its complementary sequence at different molar ratios inhibited the interaction of lnc-TSI with Smad3 *in vitro*. Data are expressed as means ± SD of three independent experiments. ∗∗∗p < 0.001.

### lnc-TSI Inhibits TGF-β1-Induced EMT in ccRCC Cells

EMT was a well-documented downstream event of TGF-β1/Smad3 pathway activation.^21^ We further evaluated the effects of lnc-TSI on TGF-β1-induced EMT in ccRCC cells. Quantitative RT-PCR and immunoblotting results showed that knocking out lnc-TSI remarkably activated EMT of ccRCC cells, including decreasing E-cadherin and increasing N-cadherin, Vimentin, and Snail in TGF-β1-stimulated ccRCC cells (Figures S2A–S2D; Figure 4A). In contrast, overexpression of lnc-TSI attenuated the TGF-β1-induced alterations of EMT markers in ccRCC cells (Figures S2E–S2G; Figure 4B). Immunofluorescence assays further demonstrated these results in Caki-1 cells (Figure 4C). To further explore the specific role of lnc-TSI on TGF-β/Smad3 signaling, we knocked down Smad3 with small interfering (siRNA) in the wild-type Caki-1 cells or cells with lnc-TSI knockout, the results of which showed that the role of lnc-TSI on EMT of Caki-1 cells was abrogated by knocking down Smad3 (Figure 4D).

**Figure 4:** lnc-TSI Inhibited TGF-β1-Induced Epithelial-Mesenchymal Transition in Caki-1 Cells (A) Representative western blot and quantitative data showed that knockout of lnc-TSI increased the expression of N-cadherin, Vimentin, and Snail and decreased the expression of E-cadherin. (B) Representative western blot and quantitative data showed that overexpression of lnc-TSI in Caki-1 cells decreased the expression of N-cadherin, Vimentin, and Snail and increased the expression of E-cadherin. (C) Immunofluorescence staining for E-cadherin and N-cadherin. (D) Representative western blot and quantitative data showed that knocking down Smad3 reversed the effects of lnc-TSI knockout. Data are expressed as means ± SD of three independent experiments. ∗p < 0.05, ∗∗p < 0.01, ∗∗∗p < 0.001.

### lnc-TSI Inhibits Invasion and Metastasis in ccRCC Cells

We analyzed whether knocking out or overexpressing lnc-TSI affects migration or invasion in ccRCC cells. Transwell assays revealed that lnc-TSI knockout enhanced ccRCC cell invasion and migration in the presence or absence of exogenous TGF-β1, and the phenomenon was more obvious upon TGF-β1 stimulation (Figure 5A; Figure S3A). Conversely, overexpression of lnc-TSI inhibited ccRCC cell invasion and migration (Figure 5B). Moreover, wound healing analysis demonstrated that the TGF-β1-induced migratory ability of Caki-1 and 786-O cells was remarkably enhanced after knocking out lnc-TSI (Figure 5C; Figure S3B), but it was inhibited by overexpression of lnc-TSI (Figure 5D). Knocking down Smad3 in lnc-TSI knockout Caki-1 cells abrogated the migration and invasion abilities enhanced by lnc-TSI knockout, indicating that the function of lnc-TSI on the migration and invasion of ccRCC cells depended on Smad3 (Figures 5E and 5F). The MTS (3-(4,5-dimethylthiazol-2-yl)-5-(3-carboxymethoxyphenyl)-2-(4-sulfophenyl)-2*H*-tetrazolium) and colony formation assays showed that there was no significant effect of knocking out or overexpressing lnc-TSI on cell proliferation (Figures S3C–S3F) and colony formations (Figures S3G and S3H) in ccRCC cells.

**Figure 5:** lnc-TSI Inhibits TGF-β1-Induced Invasion and Metastasis in ccRCC Cells (A) The representative images of Transwell assays (A_1_) and the data analysis results (A_2_–A_5_) showed that knockout of lnc-TSI enhanced cell migration and invasiveness in 786-O and Caki-1 cells compared to controls. 786-O and Caki-1 cells were treated with TGF-β1 (10 ng/mL) for 48 h. (B) The representative images of Transwell assays (B_1_) and the data analysis results (B_2_–B_5_) showed that overexpression of lnc-TSI inhibited cell migration and invasiveness in 786-O and Caki-1 cells compared to cells transfected with empty vector. 786-O and Caki-1 cells were treated with TGF-β1 (10 ng/mL) for 72 h. (C) Representative images of wound-healing assays (C_1_) and the data analysis results (C_2_ and C_3_) showed that knockout of lnc-TSI increased cell migration in both 786-O and Caki-1 cells compared to controls. (D) Representative images of wound-healing assays (D_1_) and the data analysis results (D_2_ and D_3_) showed that overexpression of lnc-TSI decreased cell migration in 786-O and Caki-1 cells compared to cells transfected with empty vector. (E) Representative images of Transwell assays (E_1_) and the data analysis results (E_2_ and E_3_) showed that knockdown of Smad3 inhibited cell migration and invasiveness induced by TGF-β1 stimulation in Caki-1 cells with or without lnc-TSI knockout. (F) Representative images of wound-healing assays (F_1_) and the data analysis results (F_2_ and F_3_) showed that knockdown of Smad3 inhibited cell migration induced by TGF-β1 stimulation in Caki-1 cells with or without lnc-TSI knockout. Data are expressed as means ± SD of three independent experiments. ∗p < 0.05, ∗∗p < 0.01, ∗∗∗p < 0.001.

### lnc-TSI Inhibits Distant Metastasis of ccRCC *In Vivo*

We then examined the biological functions of lnc-TSI in a nude mice model. lnc-TSI in luciferase-labeled Caki-1 cells were stably knocked out or overexpressed and then intravenously injected into the mice. As shown in Figure 6A, 21 days after inoculating Caki-1 cells, mice injected with lnc-TSI knockout Caki-1 cells showed remarkable bioluminescent signals in lungs, while no signals were observed in the mice injected with wild-type Caki-1 cells (Figures 6A and 6B). 60 days after inoculating Caki-1 cells, mice injected with lnc-TSI overexpressed cells had weaker bioluminescent signals compared to those injected with cells expressing empty vector (Figures 6A and 6B). The histological observations demonstrated that lnc-TSI knockout increased the metastatic lesions whereas overexpression of lnc-TSI attenuated the metastatic lesions (Figures 6C–6E). Pathological studies also confirmed these results (Figure 6F). Furthermore, immunohistochemical analysis in the lung sections collected on the 60th day after inoculation showed that the overexpression of lnc-TSI attenuated the expression of pSmad3 and the changes in EMT markers in tumor tissue from mice inoculating lnc-TSI overexpressed Caki-1 cells, as compared to the mice inoculating cells expressing empty vector (Figure 6G).

**Figure 6:** lnc-TSI Inhibited Cancer Metastasis in the Lung Metastasis Model of Nude Mice (A) Images showed the bioluminescent signal intensities of each BALB/C nude mouse after tail vein injection of Caki-1 cells treated with lnc-TSI knockout or overexpression. (B) Quantification of bioluminescent imaging signal intensities. (C) Pulmonary metastases in BALB/C nude mice after tail vein injection of Caki-1 cells treated with lnc-TSI knockout or overexpression. The arrows indicate the tumor metastases in lung. (D and E) The number (D) and the diameter (E) of the metastases in lung are shown. (F) Representative images of H&E staining and *in situ* hybridization of lnc-TSI in the lung from nude mice injected with Caki-1 cells treated with lnc-TSI knockout or overexpression. (G) Immunohistochemistry assays showed that overexpression of lnc-TSI inhibited EMT. ∗∗∗p < 0.001 (n = 6 for each group).

### The Expression Level of Tumor lnc-TSI Is Associated with Survival Rate in Patients with ccRCC

To further evaluate the expression of lnc-TSI in human ccRCC, we analyzed the expression of lnc-TSI in kidney tissue obtained at the time of radical nephrectomy from 150 patients with ccRCC. The characteristics of patients who underwent radical nephrectomy are shown in Table S1.^22^ During a 30.7-month mean follow-up, 28 patients (18.7%) passed away. The rates of tumor recurrence and metastasis information during follow-up were not available in this cohort. The expression levels of lnc-TSI in tumor tissue from patients with ccRCC were remarkably upregulated compared to the adjacent tissues by *in situ* hybridization (Figure 7A). To verify the expression of lnc-TSI in ccRCC tissue, data from the GEO ccRCC patient dataset GEO: GSE96574 were analyzed. lnc-TSI was upregulated in ccRCC tissue compared to adjacent normal tissue (Figure 7B). Furthermore, we analyzed the expression of pSmad3, N-cadherin, and E-cadherin (Figure 7C) and found that the expression level of tumor lnc-TSI was negatively correlated with pSmad3 and N-cadherin (Figures 7D and 7E) and was positively correlated with E-cadherin (Figure 7F) in ccRCC tissue. Furthermore, we found that the expression of lnc-TSI seemed higher in patients with a tumor diameter of ≤7 cm or with American Joint Committee on Cancer (AJCC) grades I and II, while the expression of lnc-TSI was comparable when these 150 patients were grouped according to their sex and age (Figures S4A–S4D).

**Figure 7:** Expression of Tumor lnc-TSI Was Associated with Survival Rate in Patients with ccRCC (A) Representative images (A_1_) of *in situ* hybridization and the data analysis results (n = 30, A_2_) showed that lnc-TSI was upregulated in human ccRCC tissues. (B) lnc-TSI was upregulated in human ccRCC tissues from GEO: GSE96574, including five-pair ccRCC tissues and adjacent normal tissues. (C) Representative images for *in situ* hybridization of lnc-TSI and immunohistochemistry assays for pSmad3, E-cadherin, and N-cadherin in tumor tissue and the adjacent normal tissue. (D–F) The Spearman’s rank correlation analysis showed associations of the lnc-TSI staining index with the pSmad3 staining index (D), N-cadherin staining index (E), and E-cadherin staining index (F) in ccRCC tissues from 150 patients with ccRCC. (G) Kaplan-Meier survival analysis showed that patients with higher expression of lnc-TSI (greater than or equal to the median) at the time of radical nephrectomy (n = 77) had a higher rate of survival during a 30.9-month mean follow-up, compared to those with lower lnc-TSI expression (below the median, n = 73). ∗∗p < 0.01, ∗∗∗p < 0.001.

We further evaluated the association between lnc-TSI expression at radical nephrectomy and survival rate during follow-up. As shown in the Kaplan-Meier analysis, the overall survival rate during follow-up was significantly better in patients with higher expression of lnc-TSI (expression index ≥ median of 5.33) compared to those with lower expression (expression index < median) at nephrectomy (p = 0.007) (Figure 7G). Cox regression analysis showed that higher expression of lnc-TSI was significantly associated with a decreased risk of all-cause death (hazard ratio [HR], 0.35; 95% confidence interval [CI], 0.15–0.79) in ccRCC patients, even after being adjusted for other cofounders such as age, sex, AJCC grade, tumor size, and node metastasis (Table 1).^22^

**Table 1:** Univariate and Multivariate Analyses of Factors Associated with All-Cause Mortality in ccRCC Patients

Variable	Univariate			Multivariate		
	HR	95% CI	p Value	HR	95% CI	p value
Age, ≤60 versus >60 years	2.50	1.18–5.29	0.016	2.28	1.03–5.08	0.061
Sex, male versus female	2.59	0.90–7.48	0.078	2.34	0.73–7.48	0.053
lnc-TSI index, ≥median versus <median	0.30	0.13–0.70	0.005	0.35	0.15–0.79	0.012
AJCC grade,^a^ >II versus ≤II	7.62	3.34–17.41	<0.001	2.94	1.08–7.99	0.056
Tumor size, >7 cm versus ≤7 cm	7.38	3.49–15.59	<0.001	7.02	3.26–15.11	<0.001
Node metastasis, yes versus no	23.49	6.29–87.76	<0.001	13.36	3.36–53.18	<0.001

CI, confidence interval; HR, hazards ratio.

a AJCC grade was defined according to the 7th edition of AJCC.^21^

## Discussion

In this study, we identified a lncRNA, lnc-TSI, which was expressed in ccRCC cells and functioned as a negative regulator for tumor metastasis. In ccRCC cells, lnc-TSI specifically inhibited the phosphorylation of Smad3 and subsequent EMT by binding with the MH2 domain of Smad3 to block the interaction between Smad3 and TβRI. lnc-TSI knockout promoted ccRCC metastasis whereas its overexpression drastically inhibited ccRCC metastasis. More importantly, in a cohort of 150 patients with ccRCC, expression levels of tumor lnc-TSI at radical nephrectomy was negatively correlated with pSmad3 and EMT markers in ccRCC tissue. Lower expression of lnc-TSI was significantly associated with a decreased risk of survival rate during follow-up, suggesting that lnc-TSI may serve as a potential therapeutic target for ccRCC.

TGF-β-induced EMT has been implicated in tumor progression and metastasis in many types of carcinomas, including ccRCC.^23^, ^24^, ^25^, ^26^ However, our understanding of the mechanism underlying the regulation of TGF-β/Smad3 signaling during cancer metastasis remains limited.^27^^,^^28^ In the present study, we provided evidence that demonstrated that lnc-TSI was an important regulator of the interaction between TβRI and Smad3 and negatively regulated TGF-β-induced EMT in ccRCC at the epigenetic and post-transcriptional levels. Consistent with our previous study in renal tubular epithelial cells,^18^ the effect of lnc-TSI was independent of other TGF-β/Smads components or regulators, such as TβRI, Sara, Smad2, Smad4, and Smad7,^29^ since there was no interaction among lnc-TSI and these components or regulators in RNA and protein interaction assay in ccRCC cells (Figure 3A). Blocking the interaction between TβRI and Smad3 specifically inhibited the phosphorylation of Smad3 and the nuclear translocation of the Smads complex, inducing subsequent EMT gene transcription in ccRCC cells. The feedback loop formed among TGF-β1, lnc-TSI, and EMT is shown in Figure S5.

ccRCC is the most common subtype of kidney cancer, and it can metastasize to various organs.^30^ An important finding in this study is that lnc-TSI may play a critical role in the metastasis of ccRCC. Previous studies have shown that the activation of TGF-β/Smads signaling promotes ccRCC metastasis in both animal models and human beings.^13^^,^^31^ Our study demonstrated for the first time that lnc-TSI inhibited ccRCC metastasis through suppressing TGF-β/Smad3 signaling. Depleting lnc-TSI enhanced ccRCC cell invasion and migration *in vitro* and attenuated ccRCC lung metastasis *in vivo*. Alternatively, overexpression of lnc-TSI inhibited ccRCC cell invasion and tumor metastasis. To further test the effect of lnc-TSI expression in human ccRCC, we analyzed lnc-TSI expression in ccRCC tissue at the time of radical nephrectomy in 150 patients with ccRCC. We found that the expression of lnc-TSI seemed higher in patients with a tumor diameter ≤7 cm or with AJCC grades I and II. However, these results need to be further confirmed due to the small sample size of patients with larger tumors or with AJCC grades III and IV in our study population. The expression of tumor lnc-TSI was correlated with the expression of pSmad3 and the alterations of EMT markers, which suggested that lnc-TSI may regulate the phosphorylation of Smad3 and subsequent EMT in human ccRCC. More importantly, patients with lower expression of tumor lnc-TSI at radical nephrectomy had lower survival rates, compared to those with higher lnc-TSI expression, during a 30.7-month mean follow-up, suggesting that the expression level of tumor lnc-TSI may predict the prognosis of patients with ccRCC.

Until now, the therapeutic design that targets the TGF-β pathway in clinical trials for cancer treatment has been focused on antibodies, antisense oligonucleotides, and kinase inhibitors for TGF-β or its receptors.^32^ Although inhibiting the TGF-β pathway results in a reduction of cancer metastasis in animal models in general, the clinical efficacy is far from satisfying. TGF-β signaling affects many physiological processes; however, these strategies may lead to adverse effects. The results of our study showed that the expression of lnc-TSI was very low in normal tubular epithelial cells and was upregulated in ccRCC cells, particularly upon TGF-β1 stimulation. lnc-TSI specifically inhibited Smad3 phosphorylation by binding with the MH2 domain of Smad3 to block the interaction between Smad3 and TβRI, suggesting that upregulation of lnc-TSI in ccRCC cells might be a self-protective mechanism for tumor metastasis and could serve as a therapeutic target. A previous study has demonstrated that inducing Smad7, a negative regulator of the TGF-β pathway, by asiatic acid, suppresses TGF-β/Smad3-mediated renal fibrosis in a mouse model.^33^ The specificity toward kidneys of lnc-TSI suggests that intervention against lnc-TSI may not affect other organs.^18^

There are limitations in this study. First, we did not evaluate the effects of lnc-TSI on other subtypes of RCC such as papillary and chromophobe, and the results may not generalize to these renal carcinomas. Second, the relationship between lnc-TSI expression and tumor metastasis or recurrence after radical nephrectomy and clinical survival analysis needs to be validated in a larger cohort study in the future.

In summary, our study showed that lnc-TSI was a critical modulator of human ccRCC metastasis. A potential molecular mechanism underlying the effect of lnc-TSI is the negative regulation of the TGF-β/Smad3-induced EMT by the inhibition of phosphorylation of Smad3 through blocking the interaction between TβRI and Smad3. lnc-TSI could serve as an independent predictor for long-term mortality in patients with ccRCC and may represent a potential therapeutic target to inhibit the metastasis of ccRCC.

## Materials and Methods

### Cell Culture

A human proximal tubular epithelial cell line (HK2) and human RCC cell lines (Caki-1 and 786-O) used in this study were commercially available (ATCC, Manassas, VA, USA). Caki-1 cells were cultured in McCoy’s 5a modified medium (Thermo Fisher Scientific, Waltham, MA, USA) supplemented with 10% fetal bovine serum (FBS) (Invitrogen, Carlsbad, CA, USA). 786-O cells were cultured in RPMI 1640 medium (Thermo Fisher Scientific). Cells were maintained at 37°C in a humidified incubator containing 5% CO_2_. For TGF-β1 stimulation, cells were serum-starved overnight when they reached 65%–75% confluence, and then they were incubated with various concentrations of recombinant human TGF-β1 (R&D Systems, USA) for the indicated time periods (Figures S1E and S1F).

### Knocking Out lnc-TSI by Using CRISPR-Cas9

To generate lnc-TSI knockout cells with CRISPR-Cas 9 gene editing, two sgRNAs targeting the gene of lnc-TSI located on chromosome 21 were cloned into U6-multiple (sgRNA)-SV40-EGFP. A Cas9-expressing vector was constructed as a Lenti-Cas9-Puro vector (GeneChem, Shanghai, China). For lnc-TSI knockout CRISPR-Cas9 clone 1, the two sgRNA sequences were as follows: sgRNA1, 5′-TTCCAGCCAGGTATCAGAGT-3′, sgRNA2, 5′-CACTGTGGGCATCTCAACCC-3′. For lnc-TSI knockout CRISPR-Cas9 clone 2, the two sgRNA sequences were as follows: sgRNA1, 5′- GAGCTAATGCTGGTGCCGTG-3′, sgRNA2, 5′-GGCTGTCGAGGCTGCAGCGA-3′. Both lentivirus-sgRNA and lentivirus-Cas9 were customized by GeneChem and applied to co-transfected target cells according to the manufacturer’s instructions.

### Overexpressing lnc-TSI

For ectopic expression of lnc-TSI, the full length of lnc-TSI cDNA was amplified by PCR and cloned into pCDH-EF1-MCS-Puro vector to generate the overexpressing plasmid. The empty pCDH-EF1-MCS-Puro vector or pCDH-EF1-MCS-Puro-lnc-TSI overexpressing vector was used to produce lentivirus in HEK293T cells with the packaging plasmids pMD2.BSBG and PSPAX2. Infectious lentiviruses were collected at 72 h after transfection of plasmids and filtered through 0.45-μm polyvinylidene fluoride (PVDF) filters. To generate lnc-TSI overexpressing ccRCCs, cells were incubated with lentiviruses and polybrene (Sigma-Aldrich, USA) followed by puromycin selection for 72 h.

### RNA Interference

For transient transfection to knock down Smad3, 50%–80% confluent Caki-1 cells were transfected with siRNA using Lipofectamine 2000 (Invitrogen) according to the manufacturer’s instructions. Sequences of siRNA (customized by GenePharma Biological Technology) targeting Smad3 were as follows: siSmad3-1, 5′-GUGAGCAGAACAGGUAGUAUUAC-3′; siSmad3-2, 5′-GAGCCUGGUCAAGAAACUCAA-3′.

### Analysis of RNA Expression

#### Real-Time PCR

Total RNA (1 μg) was extracted using TRIzol (Thermo Fisher Scientific) and reverse transcribed into cDNA using a PrimeScript RT reagent kit (Takara, Dalian, China) according to the manufacturer’s protocol. Real-time PCR was performed with a SYBR Premix Ex Taq II kit (Takara) on the LightCycler 480 system (Roche, Indianapolis, IN, USA) with the following procedure for 40 cycles: 95°C for 2 min, 90°C for 20 s, and 60°C for 1 min. The sequences of the lnc-TSI primers were 5′-AATCTGGTGTGGACAAACGC-3′ (sense strand) and 5′-AACAGATGCTTCCGAATGCC-3′ (antisense strand). The sequences of the E-cadherin primers were 5′-GCTGGACCGAGAGAGTTTCC-3′ (sense strand) and 5′-CAAAATCCAAGCCCGTGGTG-3′ (antisense strand). The sequences of the N-cadherin primers were 5′-ATGGGAAATGGAAACTTGATGGC-3′ (sense strand) and 5′-CAGTTGCTAAACTTCACTGAAAGG-3′ (antisense strand). The sequences of the Vimentin primers were 5′-GACGCCATCAACACCGAGTT-3′ (sense strand) and 5′-CTTTGTCGTTGGTTAGCTGGT-3′ (antisense strand). The sequences of the Snail primers were 5′-TCGGAAGCCTAACTACAGCGA-3′ (sense strand) and 5′-AGATGAGCATTGGCAGCGAG-3′ (antisense strand). The sequences of the β-actin primers were 5′-TGAAGTGTGACGTGGACATC-3′ (sense strand) and 5′-GGAGGAGCAATGATCTTGAT-3′ (antisense strand). The relative expression of lnc-TSI was normalized by β-actin and calculated using the CT method (2^−ΔΔCT^).

To detect the location of lnc-TSI, the nuclear and cytoplasmic fractions of ccRCCs were isolated with a Paris kit (Thermo Fisher Scientific) according to the manufacturer’s instructions. RT-PCR was performed with the separated nuclear and cytoplasmic fractions.

#### FISH

Cells were fixed in 4% formaldehyde at room temperature for 15 min. Then, the cells were permeabilized in PBS containing 0.5% Triton X-100 for 10 min on ice. Applying the digoxigenin (DIG)-conjugated oligodeoxynucleotide probes (Exiqon, Vedbaek, Denmark) for lnc-TSI and U6, hybridization was performed in hybridization solution (probes dilution 1:1,000) (Boster, Wuhan, China) overnight at 52°C in a humidified chamber. After hybridization, cells were washed in 2× standard saline citrate (SSC) for 10 min at 52°C, and then in 50% deionized formamide/2× SSC at 52°C for 30 min. The target RNA was detected with fluorescein-conjugated antibody against DIG (Roche) overnight at 4°C. Finally, the nuclei were counterstained with 4′,6-diamidino-2-phenylindole (DAPI) dihydrochloride and images were obtained by a confocal laser-scanning microscope (Carl Zeiss, Germany).

#### *In Situ* Hybridization

Paraffin-embedded tissue sections were dewaxed and rehydrated followed by digestion with trypsin (ZSGB-Bio, Beijing, China) and fixation in 4% paraformaldehyde. A DIG-labeled locked nucleic acid (LNA)-modified lnc-TSI probe (Exiqon) was diluted in hybridization solution (Boster) to create a final concentration of 25 nM. The sections were hybridized with the diluted probe at 52°C for 16 h. After extensive washing, sections were incubated with anti-DIG monoclonal antibody (Abcam, Cambridge, UK) overnight at 4°C and then dyed with nitro blue tetrazolium/5-bromo-4-chloro-3-indolylphosphate (Beyotime, China). The staining index of lnc-TSI was calculated based on the intensity and proportion of lnc-TSI-positive cells in three random fields under a ×40 objective. The proportion of positively stained cells in each field was graded as follows: 0, no positive cells; 1, ≤25%; 2, 26%–50%; 3, 51%–75%; and 4, >75%. The staining intensity of positive stained cells in each field was recorded as follows: 0, no staining; 1, light blue; 2, blue; and 3, dark blue. The staining index for each field was determined as follows: staining index = staining intensity × proportion grade of positively stained cells. The final staining index for each case was the average of the three random fields.

#### Northern Blot

Northern blots were performed using a DIG luminescent detection kit (Roche) according to the manufacturer’s instructions. Briefly, total RNA (2 μg) was mixed with RNA loading buffer (no. 9168, Takara) and heated at 65°C for 10 min. After cooling on ice for 10 min, the samples were loaded on an agarose (1.5%)-formaldehyde (2.2 M) gel at 60 V for 4 h. The separated RNAs were then transferred to a positively-charged nylon membrane (Thermo Fisher Scientific) and crosslinked with UV light. DIG-labeled LNA-modified probes (Exiqon) complementary to the target genes were hybridized to the membrane at 55°C overnight. The sequences of the probes were as follows: lnc-TSI, 5′-ACATCTCTTAATCAGCGAATCA-3′; ACTB, 5′-CTCATTGTAGAAGGTGTGGTGCCA-3′.

### Tumor Samples from Patients with ccRCC

The human ccRCCs tissue microarray (HKidE180Su02), which included 150 carcinoma tissues and 30 matched adjacent non-tumor tissues, their clinical data at time of radical nephrectomy, and the mortality during a mean of 30.7 months of follow-up, were provided by Shanghai Outdo Biotech (Shanghai, China). All patients consented to an Institutional Review Board-approved protocol that allowed comprehensive analysis of discarded tumor samples (Ethics Committee of Shanghai Outdo Biotech).

### Luciferase Reporter Assay

To determine whether lnc-TSI was transcribed by Smad3, we cloned the promoter of lnc-TSI between −1 and −2000 into the pGL3-enhancer vector (Merck Millipore, Bedford, MA, USA). Caki-1 cells were transiently transfected with pRL-TK-Renilla luciferase plasmid and pGL3-enhancer carrying lnc-TSI promoter. After 24 h, cells were collected and luciferase activity was measured with the Dual-Luciferase reporter assay system (Promega, Madison, WI, USA) according to the manufacturer’s instructions. Firefly luciferase activity was divided by Renilla luciferase activity in every sample to determine the transfection efficiency that was used to normalize the data.

### ChIP Assay

A ChIP assay was performed using a Magna ChIP HiSens chromatin IP kit (Merck Millipore) according to the manufacturer’s instructions. Caki-1 cells pretreated with TGF-β1 (10 ng/mL) for 2 h were fixed with 1% formaldehyde for 10 min at 37°C. The fixed cells were quenched with glycine and collected for sonication in an ultrasonic cell disruptor (Diagenode, Belgium) to generate DNA fragments ranging from 300 to 600 bp. IPs were performed with an antibody against Smad3 (Cell Signaling Technology, Boston, MA, USA). The binding of the promoter region of lnc-TSI to immunoglobulin G (IgG) or Smad3 was quantified using real-time PCR. Precipitated DNA fragments were detected with specific primers as follows: sense, 5′-ACAGACGGGAGTCGAGTGTA-3′, antisense, 5′-CAGACATGGGCAATCCCACT-3′.

### CoIP Assay

Cells were lysed in IP lysis buffer (Thermo Fisher Scientific) containing protease inhibitors. Cell lysates were immunoprecipitated by anti-Smad3 (Cell Signaling Technology). The immunoprecipitated complexes were captured by protein A magnetic beads (Thermo Fisher Scientific) on a magnet. After washing five times with IP lysis buffer, the immunoprecipitated proteins were separated by SDS-PAGE and detected by western blot.

### RNA Pull-Down

The full length of lnc-TSI cDNA was amplified by PCR, the complementary sequence or the delete mutations of lnc-TSI and LacZ cDNA were synthesized (Generay Biotech, Shanghai), and each sequence was cloned into the pcDNA3.1 vector (Thermo Fisher Scientific). Stem-loop A delete mutation was conducted by deleting the nt 310–333 of lnc-TSI. Stem-loop B delete mutation was conducted by deleting the nt 338–412. Stem-loop C delete mutation was conducted by deleting the nt 451–534. Biotin-labeled RNAs were transcribed *in vitro* using a MEGAscript T7 high-yield transcription kit (Thermo Fisher Scientific), labeled with biotin using a magnetic RNA-protein pull-down kit (Thermo Fisher Scientific) according to the manufacturer’s instructions. Briefly, 5 pmol of biotin-labeled RNA in RNA structure buffer (10 mM Tris [pH 7], 0.1 M KCl, 10 mM MgCl_2_) was heated at 95°C for 2 min, put on ice for 3 min, and then left at room temperature for 30 min for proper RNA secondary structure formation. Folded RNA (5 μg) was mixed with ccRCC cell lysates (5 mg) in 500 μL of Pierce IP lysis buffer (Thermo Fisher Scientific) and incubated at room temperature for 2 h. After gentle washing, streptavidin magnetic beads (50 μL) were added to each sample and incubated for 1 h. Finally, beads were washed carefully with IP lysis buffer five times and boiled in 1× loading buffer. The retrieved proteins were detected by western blot.

To determine which domain of Smad3 binds lnc-TSI, the full-length or truncated fragments sequence was separately cloned into a pCDH-CMV-EF1 (Transheep, Shanghai, China) construct with a FLAG tag at the N terminus. Caki-1 cells were transfected with plasmids carrying either the truncated fragments or the full length of Smad3. RNA pull-down was conducted on the transfected cells with biotin-labeled lnc-TSI as described above.

To determine whether the complementary sequence to lnc-TSI inhibits the interaction of lnc-TSI with Smad3, the complementary sequence of lnc-TSI was transcribed *in vitro* as mentioned above. Then, the complementary sequence and biotin-labeled lnc-TSI at different molar ratios in RNA structure buffer were heated at 95°C for 2 min, put on ice for 3 min, and then left at room temperature for 30 min for proper RNA secondary structure formation and interaction. RNA pull-down was performed as mentioned above after lnc-TSI was preincubated with its complementary sequence.

### Western Blot

The extracted proteins were separated by 10%–12% SDS-PAGE, transferred to PVDF membranes (Merck Millipore), and probed with primary antibodies against Smad2 (Cell Signaling Technology), Smad3 (Cell Signaling Technology), Smad4 (Merck Millipore), pSmad2 (Cell Signaling Technology), pSmad3 (Cell Signaling Technology), Lamin A/C (Cell Signaling Technology), SARA (Santa Cruz Biotechnology, USA), TβRI (Santa Cruz Biotechnology), β-actin (Santa Cruz Biotechnology), E-cadherin (Cell Signaling Technology), N-cadherin (Cell Signaling Technology), Vimentin (Cell Signaling Technology), and Snail (Cell Signaling Technology). After incubating with secondary antibodies, the antigen-antibody reactions were visualized using an enhanced chemiluminescence reagent (Thermo Fisher Scientific).

To detect the location of the Smads complex, the nuclear and cytoplasmic fractions of ccRCC cells were isolated with a Paris kit (Thermo Fisher Scientific) according to the manufacturer’s instructions. Western blot was performed with the separated nuclear and cytoplasmic fractions.

### Immunofluorescence Staining

Cells were fixed in 4% formaldehyde, permeabilized with 0.5% Triton X-100, and probed with the specific primary antibodies against Smad3 (Cell Signaling Technology), N-cadherin (Cell Signaling Technology), and E-cadherin (Cell Signaling Technology) overnight at 4°C, followed by incubation with secondary antibody conjugated with Alexa Fluor 488 or Alexa Fluor 594 (Invitrogen). The nuclei were counterstained with DAPI. Actin filaments were stained with DyLight 594 phalloidin (Cell Signaling Technology). Images were obtained using confocal microscopy (Leica Microsystems, Germany). To quantitatively evaluate the nuclear translocation of Smad3, cells with positive nuclear Smad3 staining were calculated in 10 random fields under a ×40 objective, and then the quantity for each sample was summed up. To analyze the co-localization of lnc-TSI and Smad3, 786-O cells were subjected to a FISH assay, then fixed for 15 min in 4% formaldehyde and subjected to immunofluorescence staining.

### Immunohistochemistry

Paraffin-embedded tissue sections were dewaxed and rehydrated followed by inhibiting endogenous peroxidase with hydrogen peroxide (3%). The slides were incubated overnight at 4°C with primary antibodies against pSmad3 (ab52903, Abcam), E-cadherin (Cell Signaling Technology), N-cadherin (Cell Signaling Technology), Vimentin (Cell Signaling Technology), and TGF-β1 (Santa Cruz Biotechnology). After extensive washing with PBS buffer, the slides were stained by an EnVision/horseradish peroxidase (HRP) kit (Dako, Denmark). The staining index for pSmad3, E-cadherin, and N-cadherin in human ccRCC samples was calculated based on the intensity and proportion of positive cells in three random fields under a ×40 objective. The proportion of positively stained cells in each field was graded as follows: 0, no positive cells; 1, ≤25%; 2, 26%–50%; 3, 51%–75%; and 4, >75%. The staining intensity of positive stained cells in each field was recorded as follows: 0, no staining; 1, light brown; 2, brown; and 3, dark brown. The staining index for each field was determined as follows: staining index = staining intensity × proportion grade of positively stained cells. The final staining index for each case was the average of the three random fields.

### Colony Formation Assay

Cells were seeded into six-well plates at a concentration of 1,000 cells per well and incubated for 7 days until colonies were clearly formed. Then, the cells were fixed and stained with 0.5% crystal violet solution. Colonies containing >50 cells were counted.

### MTS Assay

Cells were seeded into 96-well plates at a concentration of 200 cells per well and incubated for the indicated time points. Then 20 μL of MTS solution (Promega) was added to each well, followed by incubation at 37°C for 1 h. The absorbance at 490 nm was quantitatively measured in a microplate reader (BioTek, Winooski, VT, USA).

### Wound-Healing Assay

ccRCCs cells were seeded in six-well plates and grown to confluence. The adherent cells were scraped using a pipette tip to create a scratch, washed with PBS twice, and the medium was replaced with serum-free medium. Images were captured at 0, 24, and 48 h after the initial scratch and the widths of scratches were measured.

### Transwell Migration Assay

To assay the migration ability of ccRCC cells, a cell suspension containing 1 × 10^5^ cells in serum-free medium was added to the upper inserts of the Transwell migration chambers (Becton Dickinson, USA). For TGF-β1 stimulation, TGF-β1 was added to the medium of the upper inserts to make a final concentration of 10 ng/mL. The lower chambers were filled with 500 μL of culture medium supplemented with 10% FBS. Cell mobility was detected after the indicated incubation period, and cells were fixed and stained with 0.1% crystal violet. The cells that penetrated the membrane were counted in five random fields.

### Matrigel Transwell Assay

The upper inserts of the Transwell migration chambers (BD) were pre-coated with 50 μL of Matrigel (Thermo Fisher Scientific) overnight at 4°C. Then, 200 μL of cell suspension containing 1 × 10^5^ cells in serum-free medium was added to the upper inserts of the Transwell migration chambers (BD, USA). For TGF-β1 stimulation, TGF-β1 was added to the medium of the upper inserts to make a final concentration of 10 ng/mL. The lower chambers were filled with 500 μL of culture medium supplemented with 10% FBS. After the indicated incubation period, cells were fixed and stained with 0.1% crystal violet. The cells penetrated the Matrigel, and membranes were counted in five random fields.

### Xenografts

All animal experiments were approved by the Sun Yat-sen University Laboratory Animal Care and Use Committee. Male BALB/C nude mice (3-4 weeks old) were purchased from Vital River Laboratories (Beijing, China) and applied for experimental lung metastasis experiments. Caki-1 cells with lnc-TSI overexpressed or knocked out were transfected with luciferase reporter plasmid (Yeasen, Shanghai) and elected by G418 (200 μg/mL). 2 × 10^6^ cells in 200 μL of PBS were injected into the mice via the tail vein. The mice were imaged 21 days or 2 months later with luciferase-based bioluminescent imaging and analysis system (*in vivo* imaging system [IVIS] 200; Xenogen, Alameda, CA, USA) after injection of 100 μL of d-luciferin (15 mg/mL) (Yeasen, Shanghai) 10 min before imaging. After imaging, lungs were harvested from euthanized mice and fixed in paraformaldehyde for the subsequent experiments.

### Statistical Analysis

Continuous variables are expressed as means ± SD. Categorical variables are shown as numbers (percentages). Data were tested for normality using the Kolmogorov-Smirnov test. To compare normally distributed continuous variables, we conducted a two-tailed Student’s t test or one-way ANOVA with a Tukey’s *post hoc* test. To compare variables that were not normally distributed, we conducted the Mann-Whitney U test. Spearman’s rank correlations were applied for analyzing the associations between lnc-TSI expression and pSmad3 or the EMT marker expression. Kaplan-Meier survival analysis was used to demonstrate the prognostic relevance of lnc-TSI in a univariate analysis. Cox proportional hazards regression analysis was applied to analyze the independent factors on the survival prognosis of patients with ccRCC. p <0.05 was considered statistically significant.

## Author Contributions

P.W., W.C., and T.M. performed the experiments, analyzed the data, and drafted the manuscript. Z.L. and C.L. assisted with the experiments. Y.L. provided suggestions to the study design and writing of the paper. F.F.H. designed and financed the study and wrote and edited the manuscript. All authors approved the final manuscript.

## Conflicts of Interest

The authors declare no competing interests.

## Supplemental Information

Document S1. Figures S1–S5 and Table S1

Document S2. Article plus Supplemental Information

## References

[1] Greenlee R.T., Murray T., Bolden S., Wingo P.A. (2000). Cancer statistics, 2000. CA Cancer J. Clin..

[2] Siegel R.L., Miller K.D., Jemal A. (2019). Cancer statistics, 2019. CA Cancer J. Clin..

[3] Coppin C., Kollmannsberger C., Le L., Porzsolt F., Wilt T.J. (2011). Targeted therapy for advanced renal cell cancer (RCC): a Cochrane systematic review of published randomised trials. BJU Int..

[4] Frank I., Blute M.L., Cheville J.C., Lohse C.M., Weaver A.L., Leibovich B.C., Zincke H. (2003). A multifactorial postoperative surveillance model for patients with surgically treated clear cell renal cell carcinoma. J. Urol..

[5] Li P., Wong Y.N., Armstrong K., Haas N., Subedi P., Davis-Cerone M., Doshi J.A. (2016). Survival among patients with advanced renal cell carcinoma in the pretargeted versus targeted therapy eras. Cancer Med..

[6] Wang G., Zhang Z.J., Jian W.G., Liu P.H., Xue W., Wang T.D., Meng Y.Y., Yuan C., Li H.M., Yu Y.P. (2019). Novel long noncoding RNA OTUD6B-AS1 indicates poor prognosis and inhibits clear cell renal cell carcinoma proliferation via the Wnt/β-catenin signaling pathway. Mol. Cancer.

[7] Thiery J.P. (2002). Epithelial-mesenchymal transitions in tumour progression. Nat. Rev. Cancer.

[8] Wang L., Yang G., Zhao D., Wang J., Bai Y., Peng Q., Wang H., Fang R., Chen G., Wang Z. (2019). CD103-positive CSC exosome promotes EMT of clear cell renal cell carcinoma: role of remote miR-19b-3p. Mol. Cancer.

[9] Blanco M.J., Moreno-Bueno G., Sarrio D., Locascio A., Cano A., Palacios J., Nieto M.A. (2002). Correlation of Snail expression with histological grade and lymph node status in breast carcinomas. Oncogene.

[10] Yang J., Mani S.A., Donaher J.L., Ramaswamy S., Itzykson R.A., Come C., Savagner P., Gitelman I., Richardson A., Weinberg R.A. (2004). Twist, a master regulator of morphogenesis, plays an essential role in tumor metastasis. Cell.

[11] Liu Y.N., Yin J.J., Abou-Kheir W., Hynes P.G., Casey O.M., Fang L., Yi M., Stephens R.M., Seng V., Sheppard-Tillman H. (2013). miR-1 and miR-200 inhibit EMT via Slug-dependent and tumorigenesis via Slug-independent mechanisms. Oncogene.

[12] Katsuno Y., Lamouille S., Derynck R. (2013). TGF-β signaling and epithelial-mesenchymal transition in cancer progression. Curr. Opin. Oncol..

[13] Zhao B., Liu L., Mao J., Zhang Z., Wang Q., Li Q. (2018). PIM1 mediates epithelial-mesenchymal transition by targeting Smads and c-Myc in the nucleus and potentiates clear-cell renal-cell carcinoma oncogenesis. Cell Death Dis..

[14] Xu J., Lamouille S., Derynck R. (2009). TGF-β-induced epithelial to mesenchymal transition. Cell Res..

[15] Heldin C.H., Miyazono K., ten Dijke P. (1997). TGF-β signalling from cell membrane to nucleus through SMAD proteins. Nature.

[16] Massagué J. (1998). TGF-β signal transduction. Annu. Rev. Biochem..

[17] Wu D., Lei H., Wang J.Y., Zhang C.L., Feng H., Fu F.Y., Li L., Wu L.L. (2015). CTRP3 attenuates post-infarct cardiac fibrosis by targeting Smad3 activation and inhibiting myofibroblast differentiation. J. Mol. Med. (Berl.).

[18] Wang P., Luo M.L., Song E.W., Zhou Z.M., Ma T.T., Wang J., Jia N., Wang G., Nie S., Liu Y., Hou F.F. (2018). Long noncoding RNA *lnc-TSI* inhibits renal fibrogenesis by negatively regulating the TGF-β/Smad3 pathway. Sci. Transl. Med..

[19] Shou J., Cao J., Zhang S., Sun R., Zhao M., Chen K., Su S.B., Yang J., Yang T. (2018). SIS3, a specific inhibitor of smad3, attenuates bleomycin-induced pulmonary fibrosis in mice. Biochem. Biophys. Res. Commun..

[20] Hofacker I.L. (2003). Vienna RNA secondary structure server. Nucleic Acids Res..

[21] Roberts A.B., Tian F., Byfield S.D., Stuelten C., Ooshima A., Saika S., Flanders K.C. (2006). Smad3 is key to TGF-β-mediated epithelial-to-mesenchymal transition, fibrosis, tumor suppression and metastasis. Cytokine Growth Factor Rev..

[22] Edge S.B., Compton C.C. (2010). The American Joint Committee on Cancer: the 7th edition of the AJCC cancer staging manual and the future of TNM. Ann. Surg. Oncol..

[23] Tang Y.N., Ding W.Q., Guo X.J., Yuan X.W., Wang D.M., Song J.G. (2015). Epigenetic regulation of Smad2 and Smad3 by profilin-2 promotes lung cancer growth and metastasis. Nat. Commun..

[24] Li J., Zou K., Yu L., Zhao W., Lu Y., Mao J., Wang B., Wang L., Fan S., Song B., Li L. (2018). MicroRNA-140 inhibits the epithelial-mesenchymal transition and metastasis in colorectal cancer. Mol. Ther. Nucleic Acids.

[25] Cheng P., Chen Y., He T.L., Wang C., Guo S.W., Hu H., Ni C.M., Jin G., Zhang Y.J. (2019). Menin coordinates C/EBPβ-mediated TGF-β signaling for epithelial-mesenchymal transition and growth inhibition in pancreatic cancer. Mol. Ther. Nucleic Acids.

[26] Li J.K., Chen C., Liu J.Y., Shi J.Z., Liu S.P., Liu B., Wu D.S., Fang Z.Y., Bao Y., Jiang M.M. (2017). Long noncoding RNA MRCCAT1 promotes metastasis of clear cell renal cell carcinoma via inhibiting NPR3 and activating p38-MAPK signaling. Mol. Cancer.

[27] Jin K., Li T., van Dam H., Zhou F., Zhang L. (2017). Molecular insights into tumour metastasis: tracing the dominant events. J. Pathol..

[28] Bellomo C., Caja L., Moustakas A. (2016). Transforming growth factor β as regulator of cancer stemness and metastasis. Br. J. Cancer.

[29] Meng X.M., Nikolic-Paterson D.J., Lan H.Y. (2016). TGF-β: the master regulator of fibrosis. Nat. Rev. Nephrol..

[30] Capitanio U., Montorsi F. (2016). Renal cancer. Lancet.

[31] Nishida J., Miyazono K., Ehata S. (2018). Decreased TGFBR3/betaglycan expression enhances the metastatic abilities of renal cell carcinoma cells through TGF-β-dependent and -independent mechanisms. Oncogene.

[32] Neuzillet C., Tijeras-Raballand A., Cohen R., Cros J., Faivre S., Raymond E., de Gramont A. (2015). Targeting the TGFβ pathway for cancer therapy. Pharmacol. Ther..

[33] Meng X.M., Zhang Y., Huang X.R., Ren G.L., Li J., Lan H.Y. (2015). Treatment of renal fibrosis by rebalancing TGF-β/Smad signaling with the combination of asiatic acid and naringenin. Oncotarget.

